The article "Phenomenological Study on the Study Experience of Part-Time Nursing Postgraduates" was retracted in 2023. Reasons: suspected computer-generated content; unreliable results or conclusions; lack of ethics approval or compliance; missing or withdrawn patient consent.

# Phenomenological Study on the Study Experience of Part-Time Nursing Postgraduates

**DOI:** 10.1155/2022/1948691

**Published:** 2022-02-23

**Authors:** Rui Xi, Yu Wang, Aoli Huang, Baojie Zhao

**Affiliations:** ^1^School of Nursing, Jinan University, Guangzhou 510630, China; ^2^The First Affiliated Hospital of Jinan University, Guangzhou 510630, China; ^3^Community Health Service Center of Jinan University, Guangzhou 510630, China

## Abstract

In this paper, we have explored the experience of studying part-time nursing master degree students and provided a basis for improving the training of domestic part-time nursing master degree students. Using phenomenological research methods, we have conducted face-to-face and semistructured interviews with 14 part-time nursing graduate students, including postgraduate motivation, obstacles, gains, and expectations after postgraduate study. Part-time nursing master's graduate students are mostly motivated by promotion, self-improvement, solving clinical problems, and role models; barriers to entry include role conflicts, time pressure, economic pressure, curriculum settings that cannot meet needs, unclear responsibilities for training process management, and personal value (cannot reflect, etc.). Study gains include enhancing scientific research confidence, stimulating learning interest, and increasing professional identity. In the training of part-time nursing master's students, we should correctly guide students' learning motivation, mobilize social support, and solve students' learning obstacles. The curriculum of part-time nursing master's students should be targeted, along with establishing a training management system jointly directed by the training unit and the employer, improving the career planning of nursing master's students, and making a good connection with the training of senior practical nurses.

## 1. Introduction

Part-time master of nursing (hereinafter referred to as part-time master of nursing) refers to the graduate students who have passed the national unified enrollment examination for master of nursing, obtained the graduate status of general higher education, completed the credits according to the requirements of the training unit, completed nursing clinical practice, and obtained the corresponding graduation certificate and degree certificate after passing the defense of master of nursing thesis. Part-time postgraduate education is a necessary supplement to higher nursing education and an important way to cultivate nursing talents in China [1]. The 13th five year plan for national nursing development (2016) [2] proposed the following: establish a nursing talent training system connecting training units and society to comprehensively improve the quality of nursing staff. The 14th five year plan (2021) [3] proposed to actively train specialized nurses and strengthen the construction of specialized nursing capacity. Part-time nursing postgraduate education is an important part of the training of specialized nurses. In 2017, China began to coordinate the management of full-time and part-time nursing postgraduate students. However, due to the different characteristics of enrollment sources between part-time and full-time nursing postgraduate students, most of the part-time students are clinical on-the-job nurses with certain practical experience; their study experience during graduate school may be different from that of full-time students. In order to understand the motivation and obstacles of part-time nursing postgraduates, this study used the method of qualitative interview to interview 14 part-time nursing postgraduates of different grades in a university in Guangdong Province. The interview results are summarized as follows.

From literature, it is not difficult to find that there are some problems in many studies, such as vague index design, incomplete index system, and overlapping between different indexes. The reason is that scholars did not determine the principles that must be followed in the selection of evaluation indexes. On the basis of fully considering the influencing factors of learning function and user experience and drawing on the existing research results, this paper puts forward the principles that should be followed in constructing the evaluation model of learning experience based on user experience, so that the evaluation model constructed in this paper can not only reflect the characteristics of the learning experience of part-time nursing postgraduates but also ensure its scientificity and rationality.

### 1.1. Scientific Principle

Scientific principle is the most important principle when constructing the enrollment evaluation model of part-time nursing postgraduates based on user experience. It mainly emphasizes that the construction of evaluation model indicators needs to be the result of the combination of theory and practice; that is, it is required when constructing the learning experience evaluation model of part-time nursing postgraduates, whether the establishment of evaluation indicators, the selection of evaluation methods, the determination of evaluation index weight, or the collection and processing of evaluation data should be based on theoretical research. At the same time, it should be combined with the current actual situation.

### 1.2. System Integrity Principle

For the study experience, there are many factors affecting the experience. Therefore, when selecting the indicators, we should first pay attention to the integrity of the indicator selection, not only to evaluate the impact of the part-time master itself. The technical indicators of subjective emotional perception and also the nontechnical indicators that affect users' subjective emotional perception, such as school participation, talent training program, and practice, are evaluated. At the same time, we should also ensure the systematicness of index selection. We should comprehensively select indicators for evaluation research based on the characteristics and functions of part time and avoid generalizing and overlapping indicators in index selection.

### 1.3. Principle of Practicality

For any evaluation model, practicability is very important. Only the evaluation model that meets the practical requirements of easy application of the evaluation system and easy collection of evaluation data can have value. Otherwise, no matter how exaggerated the description is, the evaluation model will not have any research significance. Therefore, the selection of evaluation indicators should be clear and not complicated, and the level of indicators should be reasonable but not too much or too little. At the same time, the index setting should be intuitive and easy to understand, with clear meaning, and can easily obtain data through qualitative or quantitative measurement.

In this paper, we have explored the experience of studying part-time nursing master degree students and provided a basis for improving the training of domestic part-time nursing master degree students. Using phenomenological research methods, we have conducted face-to-face and semistructured interviews with 14 part-time nursing graduate students, including postgraduate motivation, obstacles, gains, and expectations after postgraduate study. Part-time nursing master's graduate students are mostly motivated by promotion, self-improvement, solving clinical problems, and role models; barriers to entry include role conflicts, time pressure, economic pressure, curriculum settings that cannot meet needs, unclear responsibilities for training process management, and personal value Cannot reflect, etc.; study gains include enhancing scientific research confidence, stimulating learning interest, and increasing professional identity; after graduate school, I hope to become a nursing manager and improve clinical nursing quality and scientific research capabilities.

The rest of the paper is arranged as follows: In the subsequent section, the proposed method is described in detail which is followed by a detailed section on the experimental results and observations. Generalized discussion is provided which is followed by the concluding remarks section.

## 2. Proposed Methodology

Using the objective sampling method, taking the part-time nursing postgraduates of different grades in a university in Guangdong Province as the research object, firstly, the interviewees were recruited in each class group to explain the purpose of the interview, and the interviewees were required to have good language expression and communication skills. The interview time will be determined after the interviewee is determined. Finally, 14 nontotal nursing masters were interviewed, including 5 males and 9 females, 8 married (including 7 children) and 6 unmarried. There are 5 students in grade I (grade 2020), 7 students in grade II (grade 2019), and 2 students in grade III (grade 2018). The number of interviewees in the first and second years of research is based on the fact that there is no new topic when the interview content is saturated [4]. The number of students in the third year of research who can conduct face-to-face interview is limited, and only 2 cases are included in this study. See Table 1 for the basic information of the respondents.

### 2.1. Proposed Method

#### 2.1.1. Data Collection

Using the phenomenological research method in qualitative research, the researcher and the research object conducted face-to-face semistructured interviews [5, 6]. Before the interview, the purpose, procedure, time required for the interview, and the principles of confidentiality and voluntariness are explained. The interview was conducted in a quiet and undisturbed environment, including 5 in the classroom, 8 in the demonstration classroom or conference room, and 1 in the respondent's home. During the interview, personal subjective opinions were suspended, and the interviewees were encouraged to fully express their self-experience through listening, appropriate questioning, silence, and other skills. The whole interview was recorded and the behaviors and expressions of the interviewees were recorded in time. Finally, the interview time of each case is about 20–40 minutes. The interview outline was formed by the researcher through literature review and discussion with the research group. The research team consists of one chief nurse engaged in clinical nursing education and three nursing postgraduates of different grades. The research team consists of one chief nurse engaged in clinical nursing education and three nursing postgraduates of different grades. The main contents of the interview outline include learning motivation, learning obstacles, learning gains, and postreading prospects.

#### 2.1.2. Data Analysis

The seven-step analysis method of Colaizzi qualitative research [7] is adopted, as follows:

1. Within 24 hours after the interview, the interviewer repeatedly listens to the interview recording, recalls the scene during the interview, and transcribes the interview recording into a word document in combination with the physical movements and facial expressions of the research object. The unclear part of the recording shall be verified by the interviewee.
2. Find out the important expressions related to the experience of nontotal nursing master.
3. Two researchers respectively coded frequently occurring views, such as promotion, time, self-improvement, ability, curriculum, scientific research, and harvest.
4. Sort out and summarize the coded views.
5. Write a comprehensive and detailed description.
6. Summarize similar viewpoints, classify and analyze different viewpoints, and determine the theme.
7. Finally, ask the interviewee to verify the content to confirm the accuracy of the statement.

### 2.2. Quality Control

To improve the reliability and validity of this study, the following is required:

1. When selecting respondents, fully consider the representativeness of the sample in terms of age, marital status, position, and region; reflect the characteristics of part-time nursing postgraduates at all levels of readers; and try to avoid bias caused by sample selection
2. During the interview, the researcher did not express personal opinions, avoided using inductive language and any intervention, and reduced Hawthorne effect [8]
3. In order to ensure the preciseness of data analysis, the mass method is adopted for data analysis [9]
4. All original data and analysis process shall be kept

## 3. Experimental Results

### 3.1. Study Motivation

#### 3.1.1. Promotion Needs

Most respondents said that the purpose of studying for the master of part-time nursing is to ensure that it is conducive to professional title promotion on the basis of current economic income. For example, interviewee N1: “it's just to promote the nurse in charge. I've worked for five years now. I'm the head of the Department. I do no't want to give up my current job. I can support it with salary.”. N2: “if I quit my job and study, I canno't accept it. I'm used to my current job. I just want to increase my salary after promotion”. N11: “it is an inevitable trend that the promotion to vice high school still needs the promotion of academic qualifications”.

#### 3.1.2. Self-Ability Improvement

Some respondents believe that postgraduate study is to improve themselves, improve their scientific research ability and management ability, have skills, and make life more meaningful. For example, interviewee N1: “I wanted to go to graduate school when I graduated from undergraduate school, but my family economy was average and wanted to earn my own tuition, so I chose to work first”. N2: “I love learning. Learning makes me happy.”. N3: “if you want to make life more meaningful, you just want to improve yourself.” N6: “I feel that my current job is too ordinary. I do not have technical content. As a man, I do not have any skills. It's difficult to develop in this industry.” N7: “going to graduate school is to learn and how to do scientific research.” N12: “now hospitals pay more and more attention to education and scientific research. As a nursing manager, I have to be hard. I think it's a good opportunity”. N13: “with the development of nursing, if only bachelor degree or college degree, it cannot keep up with the pace of this era”.

#### 3.1.3. Solving Clinical Practice Problems

Some respondents hope to learn how to scientifically solve clinical practice problems after postgraduate study. For example, interviewee N4: “receiving graduate education can broaden our horizons and have a deeper understanding of the problems encountered in professional practice.” N8: “going to a graduate school may make a difference in solving patient care problems.” N11: “evidence-based nursing is often heard that I want to learn to solve problems with evidence”.

#### 3.1.4. Role Model

Some respondents said that going to graduate school was to set an example for children or others, while others said they were influenced by others' examples. For example, interviewee N2: “if you want to tell your child more knowledge, tell him to do it if he has ideas, and encourage him to continue learning without stopping.” N3: “I'm married and have not had a child yet. I think the more I learn, it will also serve as an example for my children in the future.” N7: “reading graduate students is to drive colleagues to give a little bit of strength, to raise their academic qualifications, we will be more happy [*sic*] awesome cooperation.” N9: “because my husband is a doctor and my parents have a high level of education, they have set a benchmark for me”.

### 3.2. Learning Disabilities

#### 3.2.1. Role Conflict

The 14 respondents had multiple roles, including graduate students, nursing workers, parents, or children. The respondents indicated that there was a conflict between work, study, and family roles. For example, interviewee N9: “I've experienced many things in this year, such as marriage, pregnancy, Graduate School, and being a specialist team leader. I think it's very difficult to balance roles.” N13: “graduation is imminent, and it is difficult to coordinate the preparation of graduation project with the family.”

#### 3.2.2. Time Conflict

Most respondents said there was a time conflict. For example, interviewee N1: “I get up early in class almost every day and come home late. Basically, I have little time to do other things.” N2: “I cannot finish a lot of work and have no time to review. I think I'm going to drop out.” N4: “I'm very busy and do not have time to finish my homework.”

#### 3.2.3. Economic Pressure

Some respondents who have just worked or studied in other places said that there was economic pressure. For example, interviewee N3: “because there is no shuttle bus due to the long journey, you can only take a free ride every time you come to class, which costs a lot of money.” N12: “compared with full-time, our tuition fees are more expensive. For people like us who have been working for a long time, the pressure is still great.”

#### 3.2.4. Insufficient Social Support

Some respondents said that they lacked social support during their postgraduate study. For example, interviewee N4 said, “my colleagues think I often rest on weekends and will have opinions.” N3 and N8 indicate that the hospital believes that it is a personal matter to study part-time master's degree in nursing, and it is not very supportive of clinical practice out of work, so it is difficult to apply. N6 said, “at the beginning of the master's degree in part-time nursing, the society does not agree with it. People around think that nurses are injecting and making beds, and they do not think it's necessary to go to graduate school”.

#### 3.2.5. The Curriculum Cannot Meet the Needs

Most respondents believe that graduate courses should be improved compared with undergraduate courses, and the course teachers and teaching methods still need to be further improved. N1 and N4 indicate that there is no significant difference with the undergraduate learning content. N3 and N4 indicate that the teacher is still teaching the content of the textbook, and there is no specific improvement in operability, which requires a lot of self-exploration. N9 indicates that the existing courses are not very suitable for part-time students, do not greatly improve the personal clinical specialty, and lack personalization. N13 indicates that the course time is scattered, and some courses have to be partially absent due to different places.

#### 3.2.6. Unclear Responsibility of Training Process Management

Some respondents said that before clinical practice and during the implementation of graduation thesis, there were problems of unclear management responsibilities and who to look for. For example, interviewee N5: “according to the requirements of the training program, part-time nursing postgraduates need to carry out off-duty clinical practice for 3–6 months. However, when going through the formalities of off-duty clinical practice, I do not know whether to find the nursing college or the hospital nursing department”. N8: “there is no clear statement on how to apply for clinical practice of 6 months off-duty in our remote places of study. I asked many departments, spent a lot of time and took a lot of twists and turns”. N7: “because my graduation project needs to collect data from two hospitals, I am overwhelmed by the issue of subject declaration attribution and ethical declaration of research in multiple hospitals, and all departments hit a wall”.

#### 3.2.7. Personal Value Cannot Be Reflected

Some interviewees said that there was no significant difference between the clinical work of nursing graduate students and nurses with other academic qualifications, which could not well reflect their personal value. For example, interviewee N4 said: “after graduation, postgraduates feel no essential difference from undergraduates and colleges”. N8 said: “the hospital thinks that nursing postgraduates should give you more money, but they do the same job. Why not find an undergraduate or junior college student.”

### 3.3. Learning Harvest

#### 3.3.1. Enhance Confidence in Scientific Research and Stimulate Interest in Learning

Some respondents said that their confidence in nursing research increased after postgraduate study and stimulated their interest in learning relevant knowledge. For example, interviewee N2 said: “after learning scientific research related courses, it can be used immediately after class, which improves self-confidence”. N6 said: “in depth study of nursing theory increases learning interest”. However, some respondents said that the guidance of scientific research practice was insufficient. For example, N3 said: “all classes are theoretical teaching, with little practical guidance, and all rely on self-study”.

#### 3.3.2. Increased Professional Identity

Some respondents said that they had increased their professional identity after graduate school. For example, N3 said: “after learning, I have more theoretical knowledge to support me, and I think it is more meaningful to be a nurse”. N5: “because I have not worked in the clinical department, I found that nursing can also play a great role through postgraduate study. I feel very proud to be a nurse”.

### 3.4. Post Reading Outlook

#### 3.4.1. Become a Care Manager

Some respondents said that the purpose of postgraduate study is to become a nursing manager. For example, N11: “I hope I can compete for the chief nurse after graduation to lead the better development of the Department”. N13: “through graduate study, you may be engaged in management, instead of blindly doing some basic clinical nursing”.

#### 3.4.2. Improve Clinical Nursing Quality and Scientific Research Ability

Improve the quality of clinical nursing: some respondents expressed the hope that after postgraduate study, they can help improve the quality of clinical nursing and scientific research ability through their own scientific research ability and knowledge, so as to drive the development of the department. N7: “I came into contact with some new things during class, and then I felt that it was very necessary in clinic. I think there is still a lack of evidence-based quality control in clinic”. N4: “because the scientific research of our institute is still relatively weak, I want to drive and establish a scientific research team of the department”. N10: “I hope my scientific research ability will be significantly improved after studying, and I can also help my students” (research ability).

### 3.5. Determination of Index Weight

Based on the above analysis of the steps of fuzzy comprehensive evaluation, this paper takes the evaluation index of university website based on user experience as the factor set U = {U1, U2,..., UN), which is evaluated by the university website based on user experience. In order to fully judge the importance of each element of the learning experience level of part-time postgraduates, this paper uses the expert scoring method to obtain expert opinions. This paper invites 20 participants to score, including 10 full-time postgraduates and part-time postgraduates. Detailed user experience based scoring is shown in Table 2 for the relative importance of the evaluation index. 20 opinions on the relative importance of the evaluation index are obtained through scoring, and the 20 digit judgment matrix is comprehensively processed by the geometric average method to obtain the comprehensive judgment matrix. In order to facilitate the processing of the judgment matrix by AHP, the comprehensive judgment matrix is standardized and rounded. The specific rounding method is as follows: the importance of each element in the judgment matrix shall be rounded. If the importance scale is less than 1, the reciprocal shall be taken first, then rounded, and then the reciprocal shall be taken

(1) $$\begin{array}{c} x=\left\{\begin{array}{cc} \left[G\right]\;, & G\geq 1,\\ \frac{1}{\left[1/G\right]}, & G<1, \end{array}\right) \end{array}$$

where *G* is the scale value of relative importance in the attribute comprehensive judgment matrix.

(I) The first-level fuzzy comprehensive evaluation adopts the weighted average fuzzy operator *m* (x, +) model for synthesis operation, and the evaluation vector of U1 experience dimension:

(2) $$\begin{array}{c} B_{1}=W_{1}{}^{*}R_{1}=\left(0.409,0.176,0.093,0.273,0.049\right){}^{*}\left(\begin{array}{ccccc} 0.05 & 0 & 0.10 & 0.3 & 0.55\\ 0.05 & 0.05 & 0.10 & 0.25 & 0.55\\ 0.05 & 0 & 0.25 & 0.25 & 0.45\\ 0.05 & 0 & 0.20 & 0.15 & 0.6\\ 0.05 & 0.05 & 0.05 & 0.35 & 0.5 \end{array}\right). \end{array}$$

After normalization, the comprehensive evaluation vector of visual experience dimension is (0.050, 0.011, 0.139, 0.248, 0.552). According to the weighted average method, the comprehensive evaluation score of experience dimension is *S*1 = 87.41.

The weight of each index calculated is shown in the following tables.

It can be seen from Figure 1 and Table 2 that the consistency ratio of judgment matrix: C.*R* = 0.448 < 1, and the weight of emotional experience on the total goal: 0.0624. It can be seen from the above calculation results that the C.R. values of all judgment matrices are less than 0.45, so all judgment matrices get satisfactory consistency results and have high acceptability.

## 4. Discussion

### 4.1. Correctly Guiding Students' Learning Motivation

The results of this study show that the motivation of nontotal nursing master includes promotion needs, self-improvement, solving clinical problems, and role model. Learning motivation refers to a dynamic tendency to trigger and maintain students' learning behavior and make it point to certain academic goals [10]. Understanding and mastering the learning motivation of part-time nursing postgraduates is conducive to effective teaching. Correctly guide students' learning motivation to noble and correct altruism, and encourage students to closely connect graduate learning with clinical practice. Adopt motivation theory to encourage students to maintain and strengthen their learning motivation.

### 4.2. Mobilizing Social Support to Solve Students' Learning Barriers

The results of this study show that students' learning barriers include role conflict, time pressure, and economic pressure. Nontotal nursing masters generally play a variety of social roles [11–13]. How to take care of the family, do a good job, and complete learning at the same time is a major problem faced by most part-time graduate students. Therefore, it is necessary to correctly coordinate the relationship between the three. For the employer, the manager shall provide necessary emotional support and work convenience such as holding exchange meetings, mutual communication between employees and the employer and timely communication and give proper care in class arrangement to ensure class time. There should be economic support policies for employees to improve their academic qualifications, such as meal allowance, transportation expenses, or tuition subsidies after employees obtain a master's degree. For training units, students' scores should be assessed and evaluated in multiple dimensions. The assessment should be included in online learning and various learning classes. It should not be limited to lectures in training units to stimulate the enthusiasm for scientific research and learning of part-time nursing masters. In addition to the necessary papers, the achievements and rewards obtained in clinical nursing work during postgraduate study should be included in the assessment content, so as to reduce the burden of postgraduate study and increase enthusiasm, holding student exchange meetings to increase the interaction and communication between full-time and part-time students and help each other. Only by providing multifaceted support for part-time nursing masters can we further improve students' job and learning satisfaction, increase the motivation of part-time graduate students, retain talents, and finally provide better nursing services to realize the win-win of employers, training units, individuals, and patients.

### 4.3. The Curriculum of Nontotal Nursing Master Should Be Targeted

For the cultivation of master of nonholistic nursing, we should consider its particularity, consider the setting of training mode, formulate courses according to the post direction after graduation, formulate personalized course training scheme, and enrich teaching methods [14–17]. At present, the training methods of part-time and full-time nursing postgraduates are the same, lacking pertinence, and the professional development direction is relatively single, which is different from the personal clinical development direction. Paying attention to personalized professional training is the development direction of part-time nursing postgraduates. With regard to course learning, there are sufficient teachers, but the postgraduate teaching methods still need to be further explored. There is an urgent need to develop a postgraduate education system different from undergraduate education. Moreover, today's teaching methods are still mainly face-to-face teaching, which has high requirements for time and space. The incomplete master of nursing is limited by time and region, resulting in the omission of some courses. Under the impact of COVID-19, a new choice has emerged. Although online education is applied under imperfect development, it will affect teaching quality to a certain extent. But if online education develops further, developing more professional teaching software and further enriching online education interaction means, it can save time and cost for the master of noncomplete nursing. Economic cost is also an option for good teaching. For example, during working hours, courses can be supplemented to reduce absenteeism caused by work, or follow today's academic conferences, online and offline simultaneously, which is more friendly to readers in different places. Such methods can further improve learning enthusiasm and learning effect [18, 19].

### 4.4. Establishing a Training Management System Jointly Responsible by the Training Unit and the Employer

The results of this study show that there is a problem of unclear management responsibility in the process of part-time graduate training. A good postgraduate management system is the basis for postgraduate nursing students [20–22]. The clinical practice of part-time master of nursing and the smooth development of graduation project are closely related to the teaching management system. Due to the dual management of the training unit and the employing unit of part-time nursing masters, in the process of postgraduate training, if the management responsibility is not clear, it is easy to lead to the phenomenon of “kicking the ball” [23, 24]. Therefore, a training management system jointly directed by the training unit and the employer should be established to solve the problems of part-time nursing masters in the process of off-duty clinical practice and graduation project.

### 4.5. Improving the Career Planning of Nursing Postgraduates and Do a Good Job in the Connection with the Training of Senior Practical Nurses

The results of this study show that the respondents hope to engage in nursing management and improve clinical nursing quality and scientific research ability after reading, but some respondents say their personal value cannot be reflected. At present, the educational background of Chinese nurses has gradually improved and the quality of nurses has greatly improved, but the development direction of clinical work has not been clearly divided, resulting in unclear career positioning and hindered the development of career planning [25–29]. Nursing staff studying for part-time nursing masters are eager to get more opportunities and development space. Employers should pay attention to hierarchical management of nursing work and hierarchical post responsibilities and development. Training units should help students clarify their personal characteristics and choose appropriate career development directions, such as senior practical nurses or nursing managers. In terms of the training of senior practical nurses, the training courses of specialized nurses are still carried out by the society or hospital, which is not in line with the graduate education. A “one-stop” training mode of senior practical nurses between the training unit and the society or hospital should be formed, which is more conducive to the development and growth of senior practical nurses in China.

## 5. Conclusion

The cultivation and development of nontotal nursing masters is an inevitable requirement of the times. Nurses have sufficient motivation, but there are still deficiencies in the cultivation and development of nontotal nursing masters, which need to be solved with the support of the whole society from top to bottom, improve the enrollment and training management process of nontotal nursing masters' units and training units, correctly guide students' learning motivation, and improve the career planning of nursing postgraduates. The combination of online education and online and offline education is a good breakthrough for improving the learning experience of part-time nursing masters.

The results of this study only come from the Nursing College of a comprehensive university. Because there are differences in the training of master of incomplete nursing in different colleges and universities in China, there is no unified standard in China; the results of this study may not fully reflect the overall picture of psychological experience during the study of master of incomplete nursing in China. Expectation：we can use richer research methods and try to use a variety of research methods to explore this phenomenon. In addition, this study is mainly discussed from the perspective of part-time master of nursing. In the next step, it is necessary to conduct research from the perspective of relevant parties of master of nursing graduate education, such as training units and employers, so as to provide multidimensional suggestions for the improvement of part-time master of nursing graduate education.

## Figures and Tables

**Figure 1:** Comparison of teaching, examination, function, technology, and emotion.

**Table 1:** Basic information of respondents (*n* = 14).

Number	Sex	Age	Marital status	Fertility	Post	Grade	Title
N1	Female	28	Unmarried	n	Clinical nurse	I	Nurse
N2	Female	32	Married	y	Clinical nurse	I	Nurse
N3	Female	29	Married	n	Clinical nurse	I	Nurse
N4	Female	34	Unmarried	n	Clinical nurse	I	Head nurse
N5	Male	29	Unmarried	n	Nursing management	I	Nurse
N6	Male	30	Married	y	Clinical nurse	II	Nurse
N7	Female	26	Unmarried	n	Clinical nurse	II	Nurse
N8	Female	27	Unmarried	n	Clinical nurse	II	Nurse
N9	Female	29	Married	y	Clinical nurse	II	Nurse
N10	Female	29	Married	y	Clinical nurse	II	Nurse
N11	Female	32	Married	y	Nursing education	II	Head nurse
N12	Male	33	Married	y	Nursing management	II	Head nurse
N13	Male	31	Married	y	Clinical nurse	III	Nurse
N14	Male	28	Unmarried	n	Clinical nurse	III	Nurse

**Table 2:** Experience evaluation U judgment matrix of part-time postgraduates.

Part-time graduate student experience evaluation/U	Teaching experience/UI	Examination experience/U2	Functional experience/U3	Technology experience/U4	Emotional experience/U5	Weight/Wi
Teaching experience/U1	1	3	2	4	5	0.416
Examination experience/U2	1/3	1	112	2	3	0.161
Functional experience/U3	1/2	2	1	3	4	0.262
Technology experience/U4	1/4	1/3	1/2	1	2	0.099
Emotional experience/U5	1/5	1/4	1/3	1/2	1	0.062

## Data Availability

The datasets used during the current study are available from the corresponding author on reasonable request.
